The article "An End-to-End Lane Detection Model with Attention and Residual Block" was published in 2022. Journal: Comput Intell Neurosci.

# An End-to-End Lane Detection Model with Attention and Residual Block

**DOI:** 10.1155/2022/5852891

**Published:** 2022-04-13

**Authors:** Bo Wang, Xiaoting Yan, Deguang Li

**Affiliations:** School of Information Technology, Luoyang Normal University, Luoyang, 471934, China

## Abstract

Lane detection, as one of the most important core functions in the autonomous driving environment, is still an open problem. In particular, pursuing high accuracy in complex scenes, such as no line and multiple lane lines, is an urgent issue to be discussed and solved. In this paper, a novel end-to-end lane detection model combining the advantages of attention mechanism and residual block is proposed to address the problem. A residual block alleviates the possible gradient problem. An attention block can help the proposed model centralize on where to focus in the process of learning feature representation, which can make the model itself more sensitive to the feature representation of lane lines through convolutional operations. Additionally, the U-shaped structure with three downsampling operations preserves the image resolution and the original lane line information in the image to the greatest extent. The U-shaped structure can directly output the prediction results to eliminate many complex or unnecessary calculation processes. The experimental results on two public lane detection datasets show that the lane detection performance of the proposed model can achieve high accuracy, and the corresponding weight sizes are only 2.25 M. Finally, to further explain the effectiveness of the proposed model, the unavoidable troubles encountered in the experiment are discussed.

## 1. Introduction

Traffic accidents around the world will cause economic losses equivalent to US $600 billion every year [1]. As one of the countries with the largest population density and the most congested in the world, about 26% of cities in China are congested during commute peak hours [2–4]. Automatic driving technology can improve driving safety, improve the efficiency of the whole traffic system, and save time for users [5, 6].

In fact, the meaning of automatic driving is very simple [7]. The autonomous driving reduces the probability of tragedy caused by various road accidents caused by drivers and other human factors, improves traffic efficiency, and alleviates city's serious traffic congestion [8]. The drivers will be separated from the heavy and mechanized driving, which makes the travel easier, relaxed, and pleasant [9]. The liberated people can do what they want to do in the car. When studying artificial intelligence technology in the automotive industry, do the development of artificial intelligence and realize industrial upgrading [9, 10].

As one of the functions of the sensing module in driverless technology, lane detection plays an important role in the driving process of driverless vehicles [11, 12]. The research on lane detection algorithm has important research significance and application value [13].

Lane line recognition is mainly applied to automatic driving [14, 15]. After the lane line recognition is completed, the automatic driving (or still auxiliary driving) system can realize the active safety function and control function of vehicle lateral movement. For lane departure warning (LDW), when the vehicle deviates from the lane, the system can know and remind the driver through sound, touch, and other means to avoid triggering potential lateral collision or other risks after the vehicle crosses the line [16–18]. As regards lane keeping assistance (LKA), when the vehicle deviates from the lane, it will no longer be limited to sending an early warning message to the driver but actively control the steering wheel, correct the lateral position of the vehicle, correct the vehicle deviation back into the lane, and actively avoid lateral collision or other risks [19–21]. Lane centering control (LCC) can assist the driver to control the steering wheel, center the vehicle in the center of the lane, continuously control the vehicle to drive in the center of the lane, and cooperate with adaptive cruise [22–24]. As regards automatic lane change assistance, in the process of lane line recognition, we not only recognize the lane line of this lane but also add the lane line recognition of adjacent lanes. In this way, we can measure the transverse position of vehicles automatically changing from this lane to adjacent lanes. On this basis, we realize automatic lane change assistance [25, 26].

The research on lane line based on traditional methods has a long history [13]. This kind of methods mainly focuses on the characteristics related to lane line [12]. The feature-based lane line detection algorithm mainly extracts the color, texture, edge, direction, and shape of lane lines to achieve the purpose of lane line detection. The enhanced version of this kind of lane detection is the model-based detection algorithm. Usually, the curve model of lane lines is constructed, and the lane line is approximately regarded as a straight-line model, a high-order curve model, and so forth. Recently, with the great success of deep learning in the field of computer vision [27, 28], it is also widely used in the research of lane line detection, which brings new ideas for lane line detection [10]. More and more people apply deep learning to the task of lane line detection [15].

When the vehicle is in the automatic driving environment, an obvious phenomenon is that the feature change caused by dynamic change often makes the lane line detection based on traditional methods invalid. Lane detection algorithm based on deep learning method can alleviate the detection problems caused by environmental changes, but lane detection in complex scenes is still an open problem.

To address the problem, we propose a novel lane detection model, which is a U-shaped structure with three downsampling operations. To alleviate the possible gradient issue in the end of encoding network, a residual block is adopted. To obtain more effective feature representation from skip connection, an attention gate module is embedded into the decoding network. To sum up, the contributions of this paper are listed as follows:

1. A novel end-to-end lane detection model is proposed to resolve lane detection in complex scenes in the autonomous driving environment.
2. At the high-level stage of encoding network, a residual block may alleviate the possible gradient problem. An attention gate module is used to help the proposed model to focus on feature representation of lane lines.
3. In this paper, a large number of experimental results confirm the effectiveness of the proposed model, outperforming other state-of-the-art algorithms on the TuSimple and the Unsupervised Labeled Lane MArkerS (LLAMAS) dataset. The ablation study indicates that low-level features of lane lines learned by the attention module at the initial stage of the encoder network are important for lane detection.

## 2. Related Work

### 2.1. Traditional Methods

Hur et al. [29] designed a filter kernel to extract the edge information of lane signs and detected the lane signs through conditional random fields. The reason why the previously mentioned method can obtain better detection performance is that the lane edge information is obvious. When the edge information of the lane lines is lost more, Youjin et al. [30] used the segmentation algorithm to extract the lane edge information in this kind of scene. At this time, the lane line is determined according to the vanishing point (VP). The experimental results show that this algorithm is effective for lane line detection in the case of blocked or lost information. However, the algorithm is not good for lane line detection in dark light. Li et al. [31] obtained the missing points according to the extracted road text information. Gabor filter and Hough transform algorithm are used for boundary segmentation, which can achieve good results when the road text is clear. Chen et al. [32] extracted lane features according to different colors in the road. Aly [33] and others first used the segment segmentation algorithm to segment information from the processed features and then combined with the postprocessing technology to complete the further extraction and recognition of lane lines. Chiu et al. [34] first selected the region of interest, found the right threshold, and distinguished the boundaries of the corresponding lanes from the image according to the fixed value. Kim et al. [35] used a series of algorithms of filtering and postprocessing to detect lane lines in street and expressway scenes. Teng et al. [36] mixed a variety of elements to identify the characteristics of lane lines, including strip filter, color, and Hough transform. Then, in order to make the constructed algorithm realize real-time lane tracking, particle filter technology is adopted.

### 2.2. Deep Learning-Based Methods

Jiun Kim and Minho Lee [37] proposed a detector in which convolutional neural network is first used to extract lane features, which is mainly responsible for region of interest selection and boundary detection. Random sample consensus (RANSAC) is used for clustering. Deeplanes [38] is a classification based model, which has a more complex structure than literature [37]. However, the model requires location information before classification, which limits the application scenario of the model itself. Sermanet et al. [39] proposed a model named overfeat. The model improves the detection task of lane line by using classification, location, and detection. Seokju Lee et al. [40] proposed VPGNet network based on the VPD [41], which is composed of four branches to complete the detection of lane geometry. The biggest advantage of this model is that the improved vanishing point can guide lane line detection and road recognition. But the complex postprocessing process of VPGNet requires more computing resources, such as point set sampling, clustering, and lane regression. Yuhao Huang et al. [42] proposed a STLNet model including preprocessing, classification, and regression based on convolutional neural network and lane fitting. Preprocessing is used to extract lane features from the input images, while convolutional neural network is used to classify the boundary types, and the location of lane boundary is processed by regression technology. Finally, the lane lines are smoothed by fitting function. Riera Luis et al. [43] designed a lane parking detection system, in which mask RCNN [44] is used to detect the lane lines, and Kalman filter is used to track the lane lines. Pizzati Fabio et al. [45] detected drivable areas and road categories by improving ERFNet, in which DBSCAN was used to aggregate pixels in free space into a polygon.

Shao-Yuan Lo et al. [46] proposed a lane marking detection model based on the VGG architecture. Its encoding and decoding network is completely composed of dilated convolution, and the prediction result of the model is binary segmentation. Among them, the number one represents the lane line and zero represents the background other than the lane line. In addition, based on EDANet, the authors rethink the relationship between downsampling and spatial information [47] and propose another CNN network embedded with dilated convolution. At the same time, the authors also put forward two modules: feature size selection and digressive dilated block. To solve the problem of how to effectively obtain long-distance correlation information, influenced by literature [48], Wang Xiaolong et al. [49] proposed a learnable nonlocal operation to obtain the long-distance dependence between pixels. Finally, the effectiveness of this model is verified in the lane line detection task. Li Wenhui et al. [50] also applied nonlocal relations to attention networks to force CNN to focus on lane areas. Their experimental results verify the effectiveness of this idea. Similarly, according to the geometric properties of lanes, Zhang Jie et al. [51] proposed a multitask learning network, which divides lane line detection into two subtasks: lane region segmentation and lane boundary segmentation. The former segmented the selective regions and the latter pointed out the boundaries of lane lines. The experimental results show that this method can improve the detection performance of the model on lane lines as a whole by orderly combination and coordination of learning and segmenting feature information.

## 3. Proposed Model

In this section, we will introduce our model in detail, its overall structure is shown in Figure 1, and the parameters of the whole model are illustrated in Table 1. Our model is an end-to-end model and consists of an encoder network and a decoder network. The encoder network takes the original images collected by some sensors as the inputs and extracts the feature information by learning feature representations contained in the original images. After that, the decoder network is responsible for restoring the feature information learned by the encoding network to a degree consistent with the size of the input image.

### 3.1. Encoder Network

The encoder network is divided into two parts. The first part is mainly composed of sampling and convolution, which is responsible for feature extraction of the input image. The second part is made up of residual module and attention module, which is responsible for alleviating the possible gradient problem and helping the model pay attention to the most likely feature information of lane lines.

Suppose that the input image size is , where B represents batch normalization, C is channel number, and H and W represent the height and width, respectively, of an image. When the input image *x* is fed into the encoder network, firstly, the primary information of lane line is extracted from the input by the operation combination that is composed of sampling and convolution (named Inc in Table 1). At this time, the number of channels is increased from 3 to 16. In addition, in order to accelerate the operation speed of the proposed model and save computing resources, the size of the image is reduced to half of the input image. Thereafter, two similar combination operations are performed again for further extracting the high-level feature information of the lane lines. Moreover, the maximum number of channels is only 128 in our model at the high-level stage in encoder network. In particular, different from the classical end-to-end network model U-Net [52], the input image is only downsampled three times which retains more lane line semantic information to the greatest extent.

The feature information that has just been extracted is input into a residual block (bottleneck [53] is used in this paper), its internal structure is shown in Figure 2, and the whole process can be expressed as

(1) $$\begin{array}{c} H\left(x\right)=F\left(x\right)+x. \end{array}$$

*H*(*x*) is the desired mapping representation expected to be learned by our model. *F*(*x*) points to the actual mapping representation learned by our model with the help of a series of operations and represents the feature vectors of lane lines in this work. *x* indicates the feature information from the first part of encoder network and is added to the learned mapping representation *F*(*x*) as supplementary information. In this process (the red module in Figure 1), in addition to learning the desired mapping representation, the residual mechanism may also alleviate the possible gradient explosion and gradient disappearance caused by stacking network layers.

After that, to decrease false-positive predictions for lane lines that exhibit large shape variability, the output of residual block and the feature information extracted by the first part (from Inc to Maxpooling_Down3 in Table 1) are both entered into the attention gate block, which is used to filter the irrelevant feature information of lane lines and constructed under the influence of literature [54]. Its internal structure is shown in Figure 3.

In Figure 3, *g* is from the output of residual block, *x*^*l*^ implies the output of Maxpooling_Down3 in Table 1 (at this time, *l* = 3), *F*_*l*_ is the number of feature maps in layer 3 (at this time, its value is 128. Similarly, *F*_*g*_ is the number of output feature maps of residual block). At the beginning of attention gate, *x*^*l*^ is calculated for more accurate feature information of lane lines, the vector *g* determines what important regions should be focused on in this part of the content for which attention gate is responsible. Subsequently, additive attention defined in the following formulas is used to help the proposed model obtain the corresponding gating coefficient.

(2) $$\begin{array}{c} q_{\text{att}}^{l}=\psi^{T}\left(\sigma_{1}\left(W_{x}^{T}x_{i}^{l}+W_{g}^{T}g_{i}+b_{g}\right)\right)+b_{\psi }, \end{array}$$

(3) $$\begin{array}{c} \alpha_{i}^{l}=\sigma_{2}\left(q_{att}^{l}\left(x_{i}^{l},g_{i},\theta_{att}\right)\right). \end{array}$$

*W*_*x*_^*T*^, *W*_*g*_^*T*^, and *ψ*^*T*^ are the weight parameters generated by linear transformations on their inputs, and the linear transformations are acquired by using channel-wise 1 × 1 × 1 convolutions for the current input vectors. To a certain extent, biases *b*_*g*_ and *b*_*ψ*_ can cooperate with the weight parameters to adjust the network to bias the lane line feature information. Variable *σ*_*i*_ (*i* = 1, (2) means the activation function, *σ*_1_=max(0, *x*) is the ReLU function, and *σ*_2_=1/1+exp(−*x*_*i*,*c*_) indicates the sigmoid activation function. Variable q_(att)_ is the intermediate process representation of the formation of state *α*_*i*_^*l*^. q_(att)_ is a function composed of three variables *x*_*i*_^*l*^, *g*_*i*_, and *θ*_*att*_, where *g*_*i*_ determines what important regions should be focused on by the attention gate block, and *θ*_*att*_ is the comprehensive representation of other relevant parameters.

After the above ordered and complex calculation, we get its output, which can be expressed by the following formula:

(4) $$\begin{array}{c} {\hat{x}}_{i,c}^{l}=x_{i,c}^{l}\cdot \alpha_{i}^{l}. \end{array}$$

In the above formula, ${\hat{x}}_{i,c}^{l}$ is the output produced by the input feature maps and attention coefficients through the element-wise multiplication. Variable *α*_*i*_^*l*^ is the final attention coefficient that is expected to be utilized when generating the desired focus region. Then, to help our model learn feature information well, an activation function is adopted.

### 3.2. Decoder Network

The output of the attention block is fed into the decoder network. Firstly, continuous samplings for the output are performed to gain higher-level feature information of lane lines by convolutional operations while keeping the current resolution unchanged. Then, the feature information of different scales is input to the corresponding stage of decoder network through skip connection. At this time, the concatenation operation is used to increase the amount of sampling information. Finally, a prediction result containing the desired number of channels is output (the channel number is 2 in this work).

In particular, the final output has the same size as the input images and can directly provide the information of lane lines in the current frame. Especially, to be more practical, no postprocessing technology is used in generating the final output prediction results.

## 4. Experiments

In this section, we describe the lane detection datasets used in our experiments, explain the software and hardware platform when training, validating and testing the proposed model and other algorithms, explain the evaluation metrics corresponding to each dataset, detail the corresponding qualitative and quantitative results obtained by all models on each dataset, and specifically analyze the possible reasons for the above results.

## 5. Dataset

In this work, our model is trained, validated, and tested on two lane detection datasets: TuSimple [55] and Unsupervised LLAMAS [56], which contain different driving scenarios and correspond to different evaluation metrics.

### 5.1. TuSimple

The TuSimple dataset was released in the lane line detection challenge in 2017, aiming at training a neural network model to automatically recognize the lane lines on freeway road when a car drives. In this dataset, the training set contains 3,626 images, the verification set includes 352 images, and the test set has 2,782 images. Moreover, the resolution of each image is 1280 × 720.

The characteristics of the TuSimple dataset are as follows: (1) The number of lane lines is unevenly distributed, generally ranging from 2 to 7 and up to 8 or 9 in some scenes. (2) Some lane lines have no obvious features, such as no color difference. (3) There are many lane lines at the edge of road but relatively few labels in the corresponding ground truths.  Table 2 shows more information about TuSimple dataset.

### 5.2. Unsupervised LLAMAS

The Unsupervised LLAMAS dataset was released in 2019, aiming at providing an alternative dataset for the lane detection task. An obvious characteristic of this dataset different from other datasets is that the lane lines in each frame are marked completely by software. The specific conditions are as follows: (1) The labels corresponding to the lane lines on both sides of the current vehicle are marked with many pixels, while other lane lines are marked with few pixels. (2) The number of pixels marked on the lane lines in each frame image accounts for about 2% of the whole frame image. (3) The lane line close to the current vehicle, whether both sides or other conditions, is marked with more pixels, while the lane line far from the current vehicle is marked with only a few pixels.

In the Unsupervised LLAMAS dataset, the training set contains 58,269 images, the verification set includes 844 images, and the test set has 20,000 images. Moreover, the resolution of each image is 1276 × 717. More information is in Table 2.

### 5.3. Implementation Details

All the models in our experiments are trained, validated, and tested on a platform with an Intel Core i7-6800k CPU, 64 GB of RAM, and one NVIDIA TITAN Xp 12 GB GPU. The proposed model is implemented based on the PyTorch by using Python 3. The optimizer is the Adam function, the initial value of learning rate is 0.01, and the batch size is set to 10. The images are resized to 128 × 256 when they are entered into a model. Taking the TuSimple dataset as an example, Figures 4 and 5, respectively, show the change process of loss function and F1-Measure of our model during training, validation, and testing.

The class imbalance caused by the huge difference between lane line pixels and background pixels will affect the parameter learning in the process of training model, the weight cross entropy loss is used to balance the error between the real value and the predicted value, and its definition can be expressed as follows:

(5) $$\begin{array}{c} L_{w}\left(r,p\right)=-\log\left(\frac{\exp\left(p\left[\arg\max\left(r\right)\right]\right)}{\sum_{j}\exp\left(p\left[j\right]\right)}\right), \end{array}$$

where *r* and *p* represent the ground truth and the predicted result, respectively. The value of *r* represents the number of lane lines in the corresponding image. The *argmax* function will return the indexes of max values in a row in the corresponding ground truth. The operation of *p[j]* acquires the values which correspond to those indexes returned by *argmax* function.

### 5.4. Metrics

(6) $$\begin{array}{c} ACC=\frac{TP+TN}{N}\;, \end{array}$$

(7) $$\begin{array}{c} PRE=\frac{TP}{TP+FP}, \end{array}$$

(8) $$\begin{array}{c} REC=\frac{TP}{TP+FN}, \end{array}$$

(9) $$\begin{array}{c} F-\text{Measure}=\frac{\left(1+\beta^{2}\right)\left(\text{Precision}*\text{Recall}\right)}{\text{Precision}+\text{Recall}}, \end{array}$$

(10) $$\begin{array}{c} AP=\sum_{i}^{U}\left(\sum_{j}^{V+1}\left({\text{Precision}}_{j}*\Delta {\text{Recall}}_{j}\right)\right). \end{array}$$

For the TuSimple dataset, the metrics refer to the variables [57]: *ACC, PRE, REC,* and F-Measure, which are defined in formulas (6)–(9), respectively. For the Unsupervised LLAMAS dataset, in addition to the metrics of *PRE* and *REC*, the corresponding formula (10) is used to calculate the average precision (*AP*) [56] to evaluate the performance of a model. Variable *U* represents the total number of tests, *V* represents the number of tests on a frame, and *i* and *j* represent their corresponding change subscripts, respectively. Obviously, these formulas involve the basic variables *TP*, *TN*, *FP*, and *FN*.  Table 3 shows their detailed information.

If a pixel is already on the lane line and the pixel is also at the same position on the lane line in the prediction result, the prediction result is recorded as *TP*. However, in this paper, *TP* represents the sum of all these pixels. If a pixel is not on the lane line and the pixel is not at the same position on the lane line in the prediction result, the sum of such pixels is represented by *TN*. If a pixel is on the lane line but, in the prediction result, the pixel at the same position is not on the lane line, the sum of such pixels is taken as *FN*. If a pixel is not on the lane line but the pixel at the same position is on the lane line in the prediction result, the sum of such pixels is represented by *FP*.  Table 3 shows a more concise representation of those variables.

Given the above representation, *ACC* represents the proportion of pixels correctly predicted in all prediction results. *PRE* means the proportion of pixels correctly predicted on those lane lines in the prediction results. *REC* indicates the proportion of pixels predicted correctly on all lane lines to pixels predicted on all lane lines. F-Measure, as a comprehensive indicator to balance the metrics of *PRE* and *REC*, generally reflects the performance of a model. In this paper, *β* equals 1, and *F1-Measure* is taken for evaluating the whole performance of a model.

## 6. Results and Analysis

We first train our model on the TuSimple dataset and then validate and test it on the corresponding subdatasets of TuSimple.  Figure 6 shows the visual results of qualitative evaluation of our model and other state-of-the-art algorithms.

As can be seen from Figure 6, the test results of our model are better than those of other models. For example, in the image in column one, there are four lane lines in this scene. Although a large number of pixels are marked in the label corresponding to the leftmost and rightmost lane lines, there is very little information in the original image, which brings some difficulties to the feature learning of a model. This difficulty is also reflected in the test result diagram of a model, such as intermittent results (ENet [58]), incomplete results (LaneNet [59], SegNet [60], and SegNet_ConvLSTM [57]), or results containing a small number of interference signals (SCNN [61], U-Net, and U-Net_ConvLSTM [57]). In addition, from the test results in column two, when the curvature of the lane line is large, the test results of other models are not ideal. When facing the scene with less information in the original image and more lane lines (such as column four, there are more than 4 lane lines in the image), the test results of other models show more inadaptability. Some models (ENet, SCNN, and U-Net) only test incomplete lane lines, and some models (the rest algorithms) can test complete but unsatisfactory lane lines. For those lane lines that actually exist but are not marked in the ground truth, our model can detect them well, while other models cannot test them well.

Then, we test the quantitative results of all the models, and more information is displayed in Table 4. The *ACC* value of our model is 97.98%, which is closest to that of U-Net_ConvLSTM (98.21%). According to its formula (6), when the *ACC* value is high, we can conclude that the sum of *TN* and *TP* is relatively large. But we cannot continue to further infer whether the value of *TP* is high or the value of *TN* is high. Furthermore, we cannot explain the performance of a model according to the *ACC* value. Therefore, the value of ACC can only generally indicate whether a model is valid.

To further accurately evaluate the performance of a model, we introduce *PRE* and *REC* which work together and can finely determine the real performance of a model. For example, the *REC* value of U-Net_ConvLSTM is 0.958, which is higher than that of the proposed model. It means either the *TP* value is high or the *FN* value is low. If the *TP* value is really high, at this time, it truly reflects the effectiveness of U-Net_ConvLSTM model. On the contrary, if the *FN* value is low, it cannot accurately describe the performance of U-Net_ConvLSTM model. With the addition of metric *PRE*, the situation is completely different. When the values of *REC* and *PRE* are increased at the same time and the difference between them is small, it can be comprehensively judged that the performance of a model is better. In Table 4, the difference between *REC* and *PRE* of our model is 0.082, which is less than the difference (1.02) between *REC* and *PRE* of U-Net_ConvLSTM model. Moreover, the value of *PRE* in our model is larger than that in U-Net_ConvLSTM model, which further confirms that the value of *TP* in the test results of our model is higher and the value of *FP* is lower.

When the *TP* value in our model is high, it implies that our model can accurately predict more pixels that are originally on the lane lines. When the *FN* is low and the *FP* is also low, they, respectively, indicate that our model rarely predicts the pixels originally belonging to the lane line as the background and rarely predicts the pixels originally belonging to the background as the pixel babblers on the lane line. The above analysis confirms the validity of our model exactly and concretely, which also strongly proves why our model in Figure 6 can predict better results.

Additionally, another comprehensive metric, F1-Measure, is used to evaluate each model. To more clearly explain the evaluation of F1-Measure on model performance, we simplify its definition and show the impact of F1-Measure on key variables (*TP*, *FP*, and *FN*) in a clearer expression. In Table 4, the F1-Measure of our model is the highest, achieving 0.909. This demonstrates that the value of *(FN* *+* *FP)/TP* is small. To be exact, the value of *(FN* *+* *FP)* is relatively small. When the values of *FN* and *FP* are small, the corresponding metrics of our model are high, and the corresponding visual results are better than those of other models.

(11) $$\begin{array}{c} F1-\text{Measure}=2\times {\left(2+\frac{FN}{TP}+\frac{FP}{TP}\right)}^{-1}. \end{array}$$

We also test our model and other algorithms on the Unsupervised LLAMAS dataset; the detailed process of our model is shown in Figure 7. From the test results of each model, the following can be clearly seen: (1) Each model can detect most of the ego lines on the left and right sides of the current vehicle. The test results of LaneNet, Attention U-Net [54], SegNet, and U-Net are relatively few and incomplete. (2) Only a few models can detect other lane lines outside both sides of the current vehicle, such as PINET (32 × 16) [62], SCNN, PINET (64 × 32) [62], and our model. It is found that the detection results of our model are more uniform and the width of the detection results is closer to the ground truth. Other models can hardly detect the lane lines distributed outside the two sides of the current vehicle. (3) For the prediction of pixels on distant lane lines, only Attention U-Net, PINET (32 × 16), SCNN, PINET (64 × 32), and our model can detect them. In contrast, Attention U-Net can only detect a few pixels. Models of PINET (32 × 16), SCNN, and PINET (64 × 32) can detect slightly more than Attention U-Net, while our model can detect more.

In addition, we provide the quantitative experimental results measured on the Unsupervised LLAMAS dataset, as shown in Table 5. The *AP* value of U-Net is the highest, but its values of *PRE* and *REC* are extremely inconsistent. There is a big gap between them, and this means the model is extremely unstable on the dataset. The *AP* value can only reflect the performance of a model as a whole. Combined with its definition, the specific analysis depends on metrics *PRE* and *REC*.

For example, the *PRE* value of U-Net is 0.867, but its *REC* value is only 0.302. The imbalance between them implies that the *FN* value is very high. When the *FN* value is increased, it indicates that the U-Net model is easier to mispredict the pixels that originally belong to the lane line as the background. Therefore, we clearly see that, in the prediction results of U-Net model, there are few pixels on the corresponding lane lines. A similar situation exists in the SegNet model. In particular, the differences between *PRE* and *REC* in the models of PINET (32 × 16), SCNN, and PINET (64 × 32) achieve a good balance. It can be seen from Figure 7 that these models can predict more pixels belonging to the lane lines. However, not only are the values of *PRE* and *REC* of our model higher than the ones of those models, but also the difference between them is very small. The prediction results of our model are better than those of other models.

A large number of experimental results confirm the effectiveness of our model in the task of lane detection. The possible reasons for the above results are as follows: (1) The attention module makes the proposed model pay more attention to the local feature information of lane line by modifying the feature information from skip connection, which makes our model more sensitive to the features of lane lines. (2) In our model, the combination of attention and residual learning makes our model take computing resources on more effective feature areas at a specific stage.

### 6.1. Ablation Study

In order to further illustrate the effectiveness of the constructed model, this section discusses in detail the key problems encountered in the design process of the proposed model: (1) Which scale of lane line feature information is more important to the proposed model? (2) Is the backbone network effective for lane detection?

Consider that the attention gate module can make a model pay more attention to the more accurate local feature information. Combined with the importance of skip connection [2, 3], this paper decides embedding an attention gate module into the feature maps from the skip connection to strengthen the local feature information and then splicing and concatenating with the features of the same scale in the decoding network. In addition, in the process of designing the model, we follow the following principle: While increasing the learning feature representation of the proposed model, we should not increase the weight parameters of the model as much as possible. Therefore, we consider using an attention gate module in each layer of encoder network in our model, Tables 6 and 7, respectively, exhibit the experimental results on the TuSimple and Unsupervised LLAMAS dataset.

The experimental results imply the following: (1) In the task of lane line detection, the primary feature information is more important for our model. Therefore, when the attention gate module is used in the coded Up3, the test result of the corresponding model is the best. (2) In the advanced semantic stage of this model, the encoding structure of three downsampling operations can extract more accurate lane line feature information. Therefore, adding the attention module in the stage of Up1 cannot effectively improve the detection performance of our model on lane lines. (3) Generally speaking, all experimental results obtained on both the TuSimple and Unsupervised LLAMAS datasets confirm that when the attention gate module acts on the primary feature information of lane lines, the performance of the proposed model is improved to a certain extent.

Additionally, to further explain the effectiveness of the proposed model, an incremental experiment was performed, and the details are shown in Table 8. When embedding a combination of residual and attention block into the backbone network, the performance of the corresponding model (our model) can be improved.

## 7. Conclusion

In the complex scene of automatic driving, the pursuit of high-precision lane detection is still a difficult problem. In order to solve this problem, a novel lane detection model is designed in this paper. In order to maintain the image resolution as much as possible, the proposed model adopts three downsampling operations. In the high-level semantic stage of our model, residual operation is embedded to alleviate the possible gradient problem. In order to make more effective use of different scale feature information, the attention module with gating mechanism is used to filter the information irrelevant to the lane line feature information. Finally, the encoded content is restored to the same size as the input images through the decoding network. The experimental results show that this model with a small number of channels can detect lane lines well in complex scenes, achieve better performance compared to other lane detection models, and greatly reduce the parameters of the proposed model.

In the ablation study, by applying the gated attention module to the feature information where different skip connections from different layers are located, this paper verifies the importance of low-level feature information of lane line to this model. In addition, through the experiments on the backbone network without attention gate module and the proposed model, the results show that this model is better than the corresponding backbone network model.

In the future, the lightweight lane detection designs which can detect lane lines well in complex scenes by considering fusing more effective convolutional operations will be stidied.

## Figures and Tables

**Figure 1:** The overall architecture of the proposed model.

**Figure 2:** The internal structure of residual block.

**Figure 3:** The internal structure of attention gate.

**Figure 4:** The process of the loss change on the TuSimple dataset.

**Figure 5:** The process of the F1-Measure change on the TuSimple dataset.

**Figure 6:** Qualitative evaluation of our proposed model and other state-of-the-art deep learning models on the TuSimple dataset and all the detection results are not postprocessed. (a) Input images. (b) Ground truth. (c) ENet. (d) SCNN. (e) LaneNet. (f) SegNet. (g) SegNet_ConvLSTM. (h) U-Net. (i) U-Net_ConvLSTM. (j) Proposed model.

**Figure 7:** Qualitative evaluation of our proposed model and other state-of-the-art deep learning models on the Unsupervised LLAMAS dataset and all the detection results are not postprocessed. (a) Input images. (b) Ground truth. (c) LaneNet. (d) Attention U-Net. (e) PINET (32 × 16). (f) SCNN. (g) PINET (64 × 32). (h) SegNet. (i) U-Net. (j) Proposed model.

**Table 1:** Network architecture parameters.

Layer	Input	Output	Kernel	Stride	Padding
Inc	8 × 3 × 128 × 256	8 × 16 × 128 × 256	3	1	1
Maxpooling_Down1	8 × 16 × 128 × 256	8 × 32 × 64 × 128	3	1	1
Maxpooling_Down2	8 × 32 × 64 × 128	8 × 64 × 32 × 64	3	1	1
Maxpooling_Down3	8 × 64 × 32 × 64	8 × 128 × 16 × 32	3	1	1
Residual block	8 × 128 × 16 × 32	8 × 128 × 16 × 32			
Attention block	8 × 128 × 16 × 32	8 × 128 × 16 × 32			
Upsampling_Up1	8 × 128 × 16 × 32	8 × 64 × 32 × 64	3	1	1
Upsampling_Up2	8 × 64 × 32 × 64	8 × 32 × 64 × 128	3	1	1
Upsampling_Up3	8 × 32 × 64 × 128	8 × 16 × 128 × 256	3	1	1
Conv_1 × 1	8 × 16 × 128 × 256	8 × 2 × 128 × 256	1	1	0

**Table 2:** The information of TuSimple and Unsupervised LLMAS datasets.

Name	Train	Validation	Test	Resolution
TuSimple	3,626	352	2,782	1280 × 720
Unsupervised LLAMAS	58,269	844	20,000	1276 × 717

**Table 3:** Correspondence representation between real value and predicted value.

Real value	Predicted value	
	Positive (=1)	Negative (=0)
Positive (=1)	TP	FN
Negative (=0)	FP	TN

**Table 4:** The comparison results between our proposed model and other models on the TuSimple dataset.

Method	ACC (%)	PRE	REC	F1-Measure
ENet	97.84	0.854	0.952	0.900
SCNN	96.79	0.652	0.806	0.720
LaneNet	97.94	0.871	0.926	0.900
SegNet	97.73	0.809	0.869	0.838
SegNet_ConvLSTM	97.95	0.848	0.965	0.901
U-Net	97.91	0.861	0.945	0.902
U-Net_ConvLSTM	98.21	0.856	0.958	0.904
Proposed model	97.98	0.868	0.950	0.909

**Table 5:** The comparison results between our proposed model and other models on the Unsupervised LLAMAS dataset.

Method	AP	PRE	REC
Simple baseline	0.434	0.546	0.450
Res18-qin [53]	0.653	0.457	0.405
Res34-qin [53]	0.654	0.463	0.406
GAC Baseline1	0.778	0.748	0.307
PINET (32 × 16)	0.820	0.583	0.594
PINET (64 × 32)	0.833	0.620	0.584
LaneNet	0.816	0.418	0.701
Attention U-Net	0.819	0.415	0.702
SCNN	0.821	0.573	0.601
SegNet	0.893	0.863	0.201
U-Net	0.911	0.867	0.302
Proposed model	0.835	0.621	0.592

**Table 6:** The results of the proposed model on the TuSimple dataset when attention gate is embedded into different stages in the encoding network.

Layer	ACC (%)	PRE	REC	F1-Measure
Up1	98.15	0.8691	0.9462	0.9060
Up2	98.10	0.8683	0.9494	0.9072
Up3	97.98	0.8686	0.9507	0.9088

**Table 7:** The results of the proposed model on the Unsupervised LLAMAS dataset when attention gate is embedded into different stages in the encoding network.

Layer	AP	PRE	REC
Up1	0.8293	0.6228	0.5242
Up2	0.8282	0.6219	0.5237
Up3	0.8352	0.6214	0.5924

**Table 8:** Performance comparison of different module in proposed model on the TuSimple test dataset.

Method	ACC (%)	PRE	REC	F1-Measure
Proposed model^1^	98.08	0.8796	0.9346	0.9063
Proposed model^2^	98.12	0.8823	0.9368	0.9088

Proposed model^1^ means the model is without any residual and attention block. Proposed model^2^ indicates the model is with a residual and attention gate block.

## Data Availability

The data used to support the findings of this paper are included within the article.
